RETRACTED

# Potassium fertilization improves growth, yield and seed quality of sunflower (*Helianthus annuus* L.) under drought stress at different growth stages

**DOI:** 10.1371/journal.pone.0256075

**Published:** 2021-09-20

**Authors:** Javed Shabbir Dar, Mumtaz Akhtar Cheema, Muhammad Ishaq Asif Rehmani, Shahnwaz Khuhro, Shahjahan Rajput, Ahmad Latif Virk, Sajid Hussain, Muhammad Amjad Bashir, Suliman M. Alghanem, Fahad Mohammed Al-Zuaibr, Mohammad Javed Ansari, Kamel Hessini

**Affiliations:** 1 Department of Agronomy, SZABAC Dokri, Larkana, Pakistan; 2 School of Science and the Environment, Memorial University of Newfoundland, Corner Brook, Newfoundland and Labrador, Canada; 3 Department of Agronomy, Ghazi University, Dera Ghazi Khan, Pakistan; 4 Department of Entomology, SZABAC Dokri, Larkana, Pakistan; 5 College of Agronomy and Biotechnology, China Agricultural University, Beijing, China; 6 Institute of Hydrobiology, Chinese Academy of Science, Wuhan, China; 7 Department of Plant Protection Faculty of Agricultural Sciences, Ghazi University, Dera Ghazi Khan Punjab, Pakistan; 8 Department of Biology Faculty of Science, Tabuk University, Tabuk, Saudia Arabia; 9 Department of Botany, Hindu College Moradabad (Mahatma Jyotiba Phule Rohilkhand University Bareilly), Moradabad, India; 10 Department of Biology, College of Sciences, Taif University, Taif, Saudi Arabia; Harran Üniversitesi: Harran Universitesi, TURKEY

## Abstract

Water scarcity is a major concern for sunflower production in the semi-arid and arid regions of the world. Potassium (K) application has been found effective to alleviate the influence of drought stress; however, the impact of drought stress on seed quality of sunflower has not been reported frequently. Therefore, a field experiment was performed to determine the optimum K requirement for mitigating the adverse effects of water stress and improving growth and seed quality of spring-planted sunflower. Sunflower plants were exposed to water stress at different growth stages, i.e., I_o_ = no stress (normal irrigation), I_1_ = pre-anthesisi stress (irrigation skipped at pre-anthesis stage), I_2_ = anthesis stress (irrigation skipped at anthesis stage) and I_3_ = post-anthesis stress (irrigation skipped at post-anthesis stage). Potassium was applied at four different rates, i.e., K_o_ = 0, K_1_ = 50, K_2_ = 100 and K_3_ = 150 kg ha^-1^. The results revealed that water stress at pre- and post-anthesis stages significantly reduced plant height, head diameter, number of achenes, oleic acid contents, and phosphorus (P) uptake. However, pre-anthesis stress improved linoleic acid contents. Treatment I_o_K_3_ (stress-free with 150 kg ha^-1^ K) was optimum combination for 1000-achene weight, biological and achene yields, oil contents, protein contents, and N and P uptake. Results indicated that a higher amount of K and irrigation resulted in higher yield, whereas yield and yield components decreased with early-stage water stress. Nevertheless, potassium application lowered the impacts of waters stress compared to no application. Keeping in view these results, it is recommended that sunflower must be supplied 150 kg ha^-1^ K in arid and semi-arid regions to achieve higher yield and better seed quality.

RETRACTED

## Introduction

Suitable soil conditions, including adequate water and nutrient supply are required for optimum crop growth and yield [1–4]. Water is critical for plant metabolism at all growth stages; therefore, water stress is one of the most limiting factors for crop production in semi-arid and arid regions [5–7]. However, the impact of water stress varies depending upon the intensity and duration of stress, plant species, crop growth stage, and management practices. Certain crop growth stages (pre-anthesis, anthesis, and post-anthesis) could be more sensitive to water shortage [8–10]. Drought stress impairs protein and nucleic acid synthesis, photosynthesis and respiration, and reduces yield [10, 11]. Sunflower (*Helianthus annuus* L.) is moderately drought tolerant and successfully grows in diversified agro-climatic conditions. Sunflower has shown a positive response to irrigation in terms of growth and yield in regions with inadequate precipitation and low soil water supply [12]. Timely and judicious irrigation management, especially at critical growth stages significantly improves yield in sunflower. During its initial growth (30 days after sowing) sunflower crop merely uses 20–25% of its total crop water requirement. However, at the reproductive stage, plant requires more water, and onset of water stress can cause substantial yield losses [13, 14]. Anthesis and seed development are the most critical growth stages of sunflower to drought stress [12, 15].

Fertilizers are one of the basic inputs of agriculture and their timely availability is crucial for agricultural production [16–20]. After the introduction of high-yielding cultivars, a rapid decline has been recorded in soil nutrient status. High-yielding varieties/hybrids require higher amount of nutrients for rapid growth and high biomass accumulation [21–23]. Among macro-nutrients, potassium (K) is an essential nutrient and plays a key roles in improving crop yield and quality of the produce [15, 24]. Moreover, it strengthens crop plants by imparting resistance against drought, salinity, higher temperature, other abiotic stress, and biotic stresses including pests and diseases [4, 25–27]. Potassium contributes to the osmotic pull that draws water into plant roots; therefore, its deficiency in plants makes them susceptible to water shortage, mainly due to inability to use available water [24, 28, 29].

RETRACTED

Local production of edible oil in Pakistan is insufficient to meet the rising demands of rapidly growing population [30]. The unprecedented rate of population increase and urbanization, further widens the gap between domestic oil production and demand. Swift increase in domestic oilseed production has been the key target for economic and agricultural policymakers due to escalating import bills [31]. A wide gap is present regarding fertilizer management and irrigation requirements of sunflower crop for high seed production, better quality, and vigorous growth. Therefore, this study was conducted to assess the drought susceptibility of sunflower at different crop growth stages and mitigate drought-induced yield and quality losses by potassium application in spring-planted sunflower under semi-arid agro-climatic conditions. It was hypothesized that potassium supplementation will lower the adverse effects of drought stress on yield and seed quality of sunflower. It was further hypothesized that different growth stages will also differ in their sensitivity to drought stress. The results would help to improve the yield and seed quality of sunflower in drought-prone arid and semi-arid regions.

## Materials and methods

### Site and soil

Field experiments were performed at Agronomic Research Area, Department of Agronomy, University of Agriculture, Faisalabad, Pakistan (31.25^o^N, 73.09^o^E, and 183 m a.s.l.). The soil of research area is well-drained, sandy-clay-loam in texture (sand:silt:clay 54:24:22%) with 1.99 dSm^-1^ EC, low organic matter (1.04%), slightly alkaline (pH 8.1) with 143 and 6.24 ppm available K and P, respectively. Weather data of the experimental site during experiment was collected from Agrometeorological Unit, located at 150 m distance form the experimental site (Table 1).

**Table 1:** Monthly mean weather data for the growing season of the study during growing seasons.

	Max temp (°C)		Min. temp (°C)		Mean. temp (°C)		Rainfall (mm)		Relative humidity (%)		ET_0_ (mm)	
	1^st^ season	2^nd^ season	1^st^ season	2^nd^ season	1^st^ season	2^nd^ season	1^st^ season	2^nd^ season	1^st^ season	2^nd^ season	1^st^ season	2^nd^ season
February	20.1	27.6	9.8	13.1	14.9	20.3	35.1	14.6	67.7	52.36	1.7	2.7
March	27.8	28.2	15.3	14.6	21.6	21.4	48.6	37.1	40.8	40.7	2.8	3.2
April	35.1	37.7	18.2	20.7	26.7	29.2	10.8	0	35.5	23.4	5.7	7.1
May	38.1	42.3	23.4	27.3	30.8	34.8	18.4	24.1	31.7	23.9	7.2	8.1
June	43.3	40.3	28.7	27.1	36.1	33.7	62.5	55.6	32.5	26.2	8.7	7.9

RETRACTED

### Experimental design and treatments

Experimental treatments were arranged in randomized complete block design with split-plot arrangement with a net plot size of 3.6 m × 7.0 m and three replications. Four water stress regimes [I_0_ = control (normal irrigations), I_2_ = water stress at pre-anthesis stage (R3), I_3_ = water stress at anthesis stage (R5.5, 50% of the capitulum in anthesis), and I_4_ = water stress at post-anthesis stage (R7)] were kept in main plots, whereas potassium application rates [0 (K_0_), 50 (K_1_), 100 (K_2_) and 150 (K_3_) kg ha^-1^] were randomized in sub-plots. Sub-plots were separated by buffer zones to avoid seepage across other experimental plots.

### Crop husbandry

Before sowing, the experimental area was thoroughly irrigated, and seedbed was prepared by cultivating the soil twice, using a tractor-mounted cultivator, followed by leveling. Seeds of sunflower hybrid (‘S-278’, 3 seeds hill^-1^) were sown (10 kg ha^-1^) on February 14^th^ 2015 (season-I) and February 16^th^, 2016 (season-II) using a dibbler keeping 60 × 25 cm row × hill spacing. One plant hill^-1^ was maintained two weeks after emergence [10]. Half of the N [75 kg N ha^-1^ as urea and diammonium phosphate (DAP)] along with a full dose of phosphorous [100 kg P_2_O_5_ ha^-1^ as DAP] and potash [according to treatment, as sulfate of potash (SOP)] were soil incorporated as basal dose. The remaining nitrogen [75 kg N ha^-1^ as urea] was top-dressed at first irrigation. All agronomic practices, except K application and irrigation skipping were kept normal and uniform following local recommendations. of plant protection measures to keep the crop free from diseases, insect pests, and weeds.

### Irrigation methodology

Crop was irrigated according to treatments using a siphon tube (length = 5 m, diameter = 7.62 cm). Timing and quantity of irrigation water application were calculated using the formula described earlier [32].

T = Ad/Q

Where t denotes the time (h) of irrigation, A is field area (m^2^), d is depth (mm) of irrigation water applied and Q volume of water discharged per unit time (m^3^ sec^-1^).

Six siphon tubes were calibrated and shifted to different plots. A water control barrier was prepared at cross-channel area to control water flow. Time measurement was done with the help of a stopwatch and at a measured time (two siphon tubes take 5 min and 15 sec. for the discharge of 630 L of water) siphons were shifted to the other field.

### Measurements

Ten plants were randomly selected from each experimental unit, marked for the assessment of growth stages and used for measurement of plant height, head diameter, number of achenes head^-1^ and 1000-achene weight. The collected data were averaged for different treatments [29]. The plant population was counted at harvest. Plant height (cm) was measured by using measuring rod, from ground level to the base of capitulum. Subsequently, same plants were used for the measurement of head diameter (cm) using measuring tape. At harvest maturity, three rows (from each experimental unit) were manually harvested and crop samples were sun-dried. The weight of plants from each plot was recorded for biological yield [3]. For achene yield heads were separated and threshed manually to calculate seed yield from each experimental plot subsequently converted to hectare basis [10].

RETRACTED

Leaf area of six randomly selected plants per experimental plot was measured by using leaf area meter (Licor, Model 3100). Ratio of leaf area to the land area was used to calculate the leaf area index (LAI) [19]. Net assimilation rate (NAR) and crop growth rate (CGR) were estimated following [33] as described earlier [34].


$$\mathrm{NAR}=\frac{W_{2}‐W_{1}}{T_{2}-T_{1}}\times \frac{\ln\;{\mathrm{LA}}_{2}-\ln\;{\mathrm{LA}}_{1}}{{\mathrm{LA}}_{2}-{\mathrm{LA}}_{1}}$$

Where NAR is net assimilatin ration (g cm^-2^ day^-1^). The W_1_ and W_2_ are crop dry weights at first and second observation. T_2_-T_1_ is time difference between first and second observation. LA_2_-LA_1_ is difference in leaf area between two observations. The ln is natural logarithm.


$$\mathrm{CGR}=\frac{W_{2}‐W_{1}}{T_{2}–T_{1}}$$

Where CGR is crop growth rate (g m^-2^ day^-1^). The W_1_ and W_2_ are crop dry weights at first and second observation. T_2_-T_1_ is time difference between first and second observation.

### Achene oil and protein contents (%)

Soxhlet fat extraction method was used to determine seed oil contents by random selection of samples from the experimental units [35]. Protein contents of achenes were determined as an average of one sample from each replication by using micro-Kjeldahl method [35].

### Achene-fatty acid profile (%)

Fatty acid composition was determined using Shamadzo Gas Liquid Chromatograph (GLC), Model CS-7 with a glass column (2.1 m × 3.2 mm) packed with 3% SP2310/2% / SP2300 coated chromosorb WAW on 100/120 mesh. For the analysis, the column oven was operated at 230°C. Methylating solution (4 g metallic sodium) was used for preparing methyl esters of oil.

### Nutrient uptake

Collected plant samples (n = 144) were oven-dried (72°C to constant weight), ground using an electric grinding machine and stored in clean dry plastic bags for chemical analysis. The nitrogen contents of achenes and stalk (including stem, leaf, and head) were determined following micro-Kjeldahl method [35].

RETRACTED

Oven-dried plant materials (1 g) were digested in the di-acid mixture (10 ml of 72% HClO_4 +_ 20 ml concentrated HNO_3_) and subsequently cooled. The digest was transferred to a 100 ml volumetric flask to make volume with distilled water. Phosphorus concentration was observed on a spectrophotometer at 410 nm. For potassium, an aliquot from the digested material was taken to determine K^+^ using a flame photometer (Jenway PFP-7 Flame Photometer) equipped with a K^+^ filter (Method 58a). Phosphorus and potassium concentrations (%) in plant samples were calculated using a standard curve and then converted in plant uptake by multiply with yield.

### Statistical analysis

Collected data were statistically analyzed using MSTAT-C [36]. The overall significance of the data was evaluated using analysis of variance (ANOVA), treatment means were compared through the least significant difference (LSD) test at the 0.05 level.

## Results

Water stress at different growth stages and potassium fertilizer levels significantly influenced various growth, yield and quality parameters of sunflower. Skipping irrigation at different crop growth produced a significant effect on crop yield. Yield reduction depends on the degree of plant water stress at critical growth stages. Limited water supply is frequently associated with yield reduction. Both water stress and potassium application significantly affected head diameter and number of achenes (Table 2). Plant height was significantly affected by water stress; however, different level of potassium had no effect in this regard (Table 2). The tallest plants were recorded from normal irrigation, while the shortest plants were recorded from pre-anthesis stress. There was a non-significant effect of water stress and potassium application levels on plant population.

**Table 2:** Effect of water stress at different growth stages and potassium application on agronomic traits and yield components of sunflower.

Treatments	Plant population (m^-2^)		Plant height (cm)		Head diameter (cm)		No. of achenes head^-1^	
	1^st^ season	2^nd^ season	1^st^ season	2^nd^ season	1^st^ season	2^nd^ season	1^st^ season	2^nd^ season
**Water stress (W)**								
**I**_**0**_	166.75	167.00	164.47 a	161.67 a	20.09 a	19.48 a	1062 a	1026 a
**I**_**1**_	166.50	166.50	147.24 d	144.87 d	15.57 d	15.09 d	865 d	845 d
**I**_**2**_	166.50	166.42	156.82 c	153.20 c	16.04 c	15.78 c	935 c	906 c
**I**_**3**_	166.92	166.50	162.04 b	156.02 b	18.11 b	17.48 b	1004 b	974 b
**LSD**	**ns**	**ns**	**1.71**	**2.07**	**0.28**	**0.29**	**43**	**41**
**Potassium application levels (K)**								
**K**_**0**_	166.83	166.75	156.97	153.28	16.70 b	16.24 b	937 b	905 b
**K**_**1**_	167.00	166.42	157.59	153.89	16.75 b	16.29 b	949 b	918 b
**K**_**2**_	166.58	166.50	158.28	154.56	18.06 a	17.53 a	986 a	959 a
**K**_**3**_	166.25	167.00	157.71	154.02	18.31 a	17.77 a	993 a	970 a
**LSD**	**ns**	**ns**	**ns**	**ns**	**0.42**	**0.40**	**33**	**32**
**W × K**								
**I**_**0**_ **K**_**0**_	166.67	167.67	163.87	161.10	19.10	18.51	1022	984
**I**_**0**_ **K**_**1**_	167.33	166.33	164.26	161.49	19.24	18.65	1039	1001
**I**_**0**_ **K**_**2**_	167.00	166.67	164.80	162.03	20.89	20.25	1088	1048
**I**_**0**_ **K**_**3**_	166.00	167.33	164.85	162.07	21.15	20.49	1097	1072
**I**_**1**_ **K**_**0**_	167.33	166.33	146.66	144.30	14.88	14.42	832	813
**I**_**1**_ **K**_**1**_	166.67	166.33	146.91	144.54	15.44	14.97	845	825
**I**_**1**_ **K**_**2**_	166.33	166.33	146.82	144.46	15.74	15.25	887	866
**I**_**1**_ **K**_**3**_	165.67	167.00	148.56	146.17	16.22	15.73	896	875
**I**_**2**_ **K**_**0**_	166.67	166.00	156.37	152.75	15.69	15.44	908	875
**I**_**2**_ **K**_**1**_	167.00	166.67	156.79	153.16	15.28	15.04	915	881
**I**_**2**_ **K**_**2**_	166.33	166.00	157.72	154.06	16.49	16.22	953	931
**I**_**2**_ **K**_**3**_	166.00	167.00	156.43	152.81	16.71	16.43	959	937
**I**_**3**_ **K**_**0**_	166.67	167.00	160.97	154.98	17.12	16.57	958	948
**I**_**3**_ **K**_**1**_	167.00	166.33	162.42	156.38	17.04	16.50	997	965
**I**_**3**_ **K**_**2**_	166.67	167.00	163.78	157.68	19.12	18.40	1015	990
**I**_**3**_ **K**_**3**_	167.33	166.66	161.01	155.02	19.15	18.43	1020	994
**LSD**	**ns**	**ns**	**ns**	**ns**	**ns**	**ns**	**ns**	**ns**

I_0_ = no stress, I_1_ = pre anthesis stress, I_2_ = anthesis stress, I_3_ = post anthesis stress, K_0_ = 0 kg K ha^-1^, K_1_ = 50 kg K ha^-1^, K_2_ = 100 kg K ha^-1^, K_3_ = 150 kg K ha^-1^, LSD = least significant difference, ns = non-significant, Mean values sharing the same letter in a column do not differ significantly at P = 0.05.

RETRACTED

Head diameter and number of achene head^-1^ were significantly affected by water stress and potassium levels. Normal irrigation produced the highest number of achene head^-1^ and head diameter, while pre-anthesis stress resulted in the lowest head diameter and number of achene head^-1^. Treatment K_3_ observed the highest head diameter and number of achenes head^-1^ and these results were statistically at par with K_2_. Treatments K_0_ and K_1_ had statistically similar results, while the lowest values were recorded for K_0_.

Major yield parameters, i.e., 1000-achene weight, achene yield, and biological yield were significantly affected by the interactions among water stress and potassium application, while had non-significant effect on harvest index (Table 3). Treatment I_0_K_3_ was optimum and resulted in the highest 1000-achene weight, achene yield, and biological yield during both years.

**Table 3:** Effect of water stress at different growth stages and potassium application on 1000 achene weight, achene yield, biological yield and harvest index.

Treatments	1000-achene weight (g)		Achene yield (kg ha^-1^)		Biological yield (kg ha^-1^)		Harvest index	
	1^st^ season	2^nd^ season	1^st^ season	2^nd^ season	1^st^ season	2^nd^ season	1^st^ season	2^nd^ season
**Water stress (W)**								
**I**_**0**_	55.85 a	54.32 a	2997 a	2921 a	8311 a	8409 a	36.05 a	34.72 a
**I**_**1**_	48.44 d	47.15 d	2268 d	2184 d	7145 d	7054 d	31.75 d	30.97 d
**I**_**2**_	50.28 c	48.94 c	2548 c	2467 c	7685 c	7605 c	33.15 c	32.44 c
**I**_**3**_	52.24 b	50.72 b	2718 b	2635 b	7882 b	7936 b	34.49 b	33.20 b
**LSD**	**0.90**	**0.74**	**43**	**47**	**95**	**150**	**0.69**	**0.70**
**Potassium application levels (K)**								
**K**_**0**_	49.92 d	48.39 d	2541 d	2460 d	7688 b	7656 b	32.97 d	32.05 c
**K**_**1**_	51.14 c	49.71 c	2589 c	2511 c	7695 b	7694 b	33.58 c	32.56 b
**K**_**2**_	52.55 b	51.20 b	2684 b	2601 b	7841 a	7826 a	34.14 b	33.16 a
**K**_**3**_	53.21 a	51.84 a	2718 a	2635 a	7798 a	7832 a	34.76 a	33.55 a
**LSD**	**0.47**	**0.47**	**32**	**31**	**78**	**59**	**0.36**	**0.40**
**W× K**								
**I**_**0**_ **K**_**0**_	54.01 d	52.35 d	2872 c	2789 c	8158 b	8227 b	35.21	33.90
**I**_**0**_ **K**_**1**_	55.10 c	53.36 c	2904 c	2837 c	8124 bc	8238 b	35.76	34.44
**I**_**0**_ **K**_**2**_	56.63 b	55.32 b	3068 b	2991 b	8468 a	8577 a	36.23	34.88
**I**_**0**_ **K**_**3**_	57.61 a	56.27 a	3144 a	3066 a	8494 a	8604 a	37.01	35.64
**I**_**1**_ **K**_**0**_	47.71 j	46.44 i	2191 j	2109 j	7139 i	7048 hi	30.69	29.93
**I**_**1**_ **K**_**1**_	48.29 ij	47.00 hi	2249 ij	2165 ij	7205 i	7114 h	31.21	30.43
**I**_**1**_ **K**_**2**_	48.60 hij	47.31 hi	2297 hi	2212 hi	7154 i	7063 hi	32.12	31.23
**I**_**1**_ **K**_**3**_	49.17 ghi	47.86 gh	2336 h	2249 h	7082 i	6992 i	32.99	32.17
**I**_**2**_ **K**_**0**_	48.62 hij	47.33 hi	2460 g	2382 g	7655 gh	7493 g	32.14	31.80
**I**_**2**_ **K**_**1**_	49.73 g	48.40 g	2511 g	2431 g	7639 h	7557 fg	32.87	32.18
**I**_**2**_ **K**_**2**_	50.71 f	49.36 f	2604 f	2521 f	7754 fgh	7619 ef	33.59	33.09
**I**_**2**_ **K**_**3**_	52.06 e	50.67 e	2617 f	2534 f	7693 fgh	7752 e	34.02	32.68
**I**_**3**_ **K**_**0**_	49.27 gh	47.44 h	2640 ef	2559 ef	7802 efg	7855 d	33.84	32.58
**I**_**3**_ **K**_**1**_	51.45 ef	50.08 ef	2692 e	2609 e	7813 ef	7866 d	34.47	33.18
**I**_**3**_ **K**_**2**_	54.26 cd	52.82 cd	2766 d	2682 d	7990 cd	8045 c	34.63	33.34
**I**_**3**_ **K**_**3**_	54.00 d	52.56 cd	2775 d	2690 d	7925 de	7979 c	35.03	33.72
**LSD**	**0.94**	**0.95**	**65**	**63**	**156**	**118**	**ns**	**ns**

I_0_ = no stress, I_1_ = pre anthesis stress, I_2_ = anthesis stress, I_3_ = post anthesis stress, K_0_ = 0 kg K ha^-1^, K_1_ = 50 kg K ha^-1^, K_2_ = 100 kg K ha^-1^, K_3_ = 150 kg K ha^-1^, LSD = least significant difference, ns = non-significant, Mean values sharing the same letter in a column do not differ significantly at P = 0.05.

RETRACTED

The highest LAI was recorded on 75 DAS. Water stress significantly decreased LAI (75 DAS), while potassium application had no effect in this regard. The lowest LAI was recorded for pre-anthesis stress. During 2015, the highest LAI was recorded from I_3_ and these results were statistically similar with I_0_. During 2016, the highest values were observed from I_0_ (Fig 1).

**Fig 1:** Effect of water stress on leaf area index of sunflower during first (a) and second (b) growing seasons.

In the fatty acid profile, stearic acid and palmitic acid were not affected by water stress (Table 4). Stearic acid was significantly influenced by potassium application. Treatment K_2_ observed the highest stearic acid contents and these results are statistically similar to K_3_ during both years. The highest linoleic acid was observed under pre-anthesis stress during both years. The lowest values of linoleic acid contents were observed for normal irrigation. Linoleic acid contents were slightly changed with increasing potassium application. Only K_3_ showed statistically significant results as compared to all other treatments. Water stress significantly reduced oleic acid contents during both years.

**Table 4:** Effect of water stress at different growth stages and potassium application on fatty acid profile.

Treatments	Stearic acid (%)		Palmitic acid (%)		Linoleic acid (%)		Oleic acid (%)	
	1^st^ season	2^nd^ season	1^st^ season	2^nd^ season	1^st^ season	2^nd^ season	1^st^ season	2^nd^ season
**Water stress (W)**								
**I**_**0**_	2.04	1.96	6.05	5.97	58.94 d	56.89 c	29.89 a	31.06 a
**I**_**1**_	2.01	1.95	6.00	5.91	62.56 a	60.27 a	27.71 c	28.56 c
**I**_**2**_	2.03	1.97	6.08	6.00	61.41 b	58.73 b	28.94 b	30.02 b
**I**_**3**_	2.02	1.96	6.12	6.01	59.98 c	57.69 c	29.15 b	30.09 b
**LSD**	**ns**	**ns**	**ns**	**ns**	**0.61**	**0.88**	**0.66**	**0.54**
**Potassium application levels (K)**								
**K**_**0**_	1.99 b	1.92 b	6.04	5.98	60.10 b	57.76 c	28.04 c	28.81 c
**K**_**1**_	1.97 b	1.90 b	6.11	5.94	60.49 b	57.98 bc	28.61 bc	29.74 b
**K**_**2**_	2.09 a	2.02 a	6.03	6.01	60.63 b	58.53 b	29.11 b	30.20 b
**K**_**3**_	2.05 a	2.00 a	6.06	5.97	61.66 a	59.32 a	29.93 a	30.99 a
**LSD**	**0.04**	**0.04**	**ns**	**ns**	**0.55**	**0.59**	**0.65**	**0.74**
**W× K**								
**I**_**0**_ **K**_**0**_	2.01	1.90	5.99	5.95	58.30	56.41	28.88	29.87
**I**_**0**_ **K**_**1**_	1.96	1.86	6.14	5.92	58.96	56.87	29.27	30.51
**I**_**0**_ **K**_**2**_	2.09	2.05	6.00	6.05	58.71	56.63	30.11	31.39
**I**_**0**_ **K**_**3**_	2.09	2.05	6.08	5.97	59.78	57.67	31.31	32.48
**I**_**1**_ **K**_**0**_	2.00	1.95	5.96	5.94	62.23	60.03	27.11	27.46
**I**_**1**_ **K**_**1**_	1.95	1.88	6.03	5.88	62.06	59.87	27.71	28.73
**I**_**1**_ **K**_**2**_	2.07	1.99	5.97	5.87	62.54	60.32	27.94	28.98
**I**_**1**_ **K**_**3**_	2.03	1.98	6.05	5.96	63.40	60.88	28.09	29.07
**I**_**2**_ **K**_**0**_	1.99	1.94	6.09	6.01	61.07	58.60	28.26	29.14
**I**_**2**_ **K**_**1**_	1.98	1.93	6.16	5.99	60.99	58.08	28.75	29.89
**I**_**2**_ **K**_**2**_	2.08	2.01	6.01	6.03	61.18	58.80	29.09	30.26
**I**_**2**_ **K**_**3**_	2.06	2.00	6.05	5.98	62.40	59.43	29.64	30.81
**I**_**3**_ **K**_**0**_	1.96	1.91	6.12	6.01	58.81	56.01	27.91	28.76
**I**_**3**_ **K**_**1**_	2.00	1.95	6.12	5.98	59.96	57.10	28.72	29.85
**I**_**3**_ **K**_**2**_	2.11	2.01	6.15	6.10	60.09	58.36	29.30	30.18
**I**_**3**_ **K**_**3**_	2.02	1.97	6.06	5.98	61.05	59.29	30.68	31.59
**LSD**	**ns**	**ns**	**ns**	**ns**	**ns**	**ns**	**ns**	**ns**

I_0_ = no stress, I_1_ = pre anthesis stress, I_2_ = anthesis stress, I_3_ = post anthesis stress, K_0_ = 0 kg K ha^-1^, K_1_ = 50 kg K ha^-1^, K_2_ = 100 kg K ha^-1^, K_3_ = 150 kg K ha^-1^, LSD = least significant difference, ns = non-significant, Mean values sharing the same letter in a column do not differ significantly at P = 0.05

Interactive effect of water stress and potassium application significantly influenced N and K uptake (Table 5). Treatment I_0_K_3_ resulted in the highest uptake of N and K in the plants against the lowest in I_1_K_0_. The highest P uptake was recorded from no stress against the minimum in pre-anthesis stress (Table 5).

RETRACTED

**Table 5:** Effect of water stress at different growth stages and potassium application on nutrient uptake.

Treatments	N uptake		P uptake		K uptake	
	1^st^ Season	2^nd^ Season	1^st^ Season	2^nd^ Season	1^st^ Season	2^nd^ Season
**Water stress (W)**						
**I**_**0**_	82.59 a	81.69 a	30.11 a	29.24 a	131.78 a	134.67 a
**I**_**1**_	56.14 d	56.31 d	17.47 d	17.71 d	72.43 d	74.72 d
**I**_**2**_	65.66 c	64.87 c	20.50 c	20.39 c	91.45 c	94.46 c
**I**_**3**_	73.92 b	72.47 b	23.79 b	23.63 b	105.96 b	109.57 b
**LSD**	**2.04**	**1.93**	**1.94**	**2.01**	**3.86**	**3.89**
**Potassium application levels (K)**						
**K**_**0**_	55.86 d	55.64 d	18.57 d	18.31 d	81.52 d	83.58 d
**K**_**1**_	63.84 c	63.95 c	20.71 c	20.57 c	88.66 c	90.89 c
**K**_**2**_	77.93 b	76.67 b	25.24 b	25.09 b	111.06 b	115.01 b
**K**_**3**_	80.68 a	79.06 a	27.35 a	27.01 a	120.37 a	123.93 a
**LSD**	**1.32**	**1.38**	**1.71**	**1.61**	**4.25**	**4.37**
**W× K**						
**I**_**0**_ **K**_**0**_	66.11 fg	66.46 f	23.35	22.48	108.03 ef	109.77 e
**I**_**0**_ **K**_**1**_	73.95 e	74.46 e	26.63	25.71	112.22 de	114.02 e
**I**_**0**_ **K**_**2**_	92.80 b	90.96 b	34.16	33.47	145.36 b	149.02 b
**I**_**0**_ **K**_**3**_	97.48 a	94.90 a	36.32	35.31	161.53 a	165.79 a
**I**_**1**_ **K**_**0**_	43.97 l	44.75 k	14.16	14.22	62.34 j	63.89 I
**I**_**1**_ **K**_**1**_	52.19 k	52.47 j	15.48	15.54	64.35 j	66.44 I
**I**_**1**_ **K**_**2**_	63.31 hi	62.93 gh	19.01	19.31	78.05 hi	80.75 gh
**I**_**1**_ **K**_**3**_	65.10 gh	65.05 fg	21.22	21.73	84.98 h	87.79 g
**I**_**2**_ **K**_**0**_	53.51 k	25.90 j	15.99	16.31	74.02 i	76.85 h
**I**_**2**_ **K**_**1**_	61.29 ij	61.23 h	18.34	18.49	82.14 hi	85.50 gh
**I**_**2**_ **K**_**2**_	73.61 e	72.84 e	22.65	22.53	102.27 fg	106.29 ef
**I**_**2**_ **K**_**3**_	74.21 e	72.49 e	25.01	24.24	107.36 ef	109.19 e
**I**_**3**_ **K**_**0**_	59.84 j	58.45 i	20.77	20.18	81.70 hi	83.81 gh
**I**_**3**_ **K**_**1**_	67.92 f	67.65 f	22.36	22.56	95.92 g	97.58 f
**I**_**3**_ **K**_**2**_	81.99 d	79.94 d	25.16	25.04	118.58 d	123.91 d
**I**_**3**_ **K**_**3**_	85.92 c	83.82 c	26.84	26.72	127.63 c	132.96 c
**LSD**	**2.64**	**2.65**	**ns**	**ns**	**8.50**	**8.73**

I_0_ = no stress, I_1_ = pre anthesis stress, I_2_ = anthesis stress, I_3_ = post anthesis stress, K_0_ = 0 kg K ha^-1^, K_1_ = 50 kg K ha^-1^, K_2_ = 100 kg K ha^-1^, K_3_ = 150 kg K ha^-1^, LSD = least significant difference, ns = non-significant, Mean values sharing the same letter in a column do not differ significantly at P = 0.05

The highest crop growth rate was recorded from I_0_ during 2015 (Table 6), whereas I_0_ and I_3_ show statistically similar results during 2016. The lowest LAI was recorded from I_1_ during both the years. Treatments K_0_ and K_3_ observed the lowest and the highest crop growth rate, respectively. Net assimilation rate (NAR) showed a different pattern than other parameters. The highest NAR was recorded for I_1_. Remaining treatments were statistically similar. However, different potassium levels were statistically similar for NAR. Interactive effect of water stress and K application significantly influenced achene oil and protein contents. The highest oil and protein contents were recorded from I_0_K_3_ during both years. Treatment I_1_K_0_ produced the minimum oil and protein contents during both years (Table 6). Increasing K application significantly improved P uptake. Higher rates of K (K_3_) resulted in better P uptake during both years. Correlation coefficients between achene yield and yield components showed a significant and positive correlation during 2015 and 2016 (Table 7).

RETRACTED

**Table 6:** Effect of water stress at different growth stages and potassium application on oil contents, protein contents, crop growth rate and net assimilation rate.

Treatments	Oil contents (%)		Protein contents (%)		Crop growth rate (CGR) (g m^-2^ day^-1^)		Net assimilation rate (NAR) (g cm^-2^ day^-1^)	
	1^st^ season	2^nd^ season	1^st^ season	2^nd^ season	1^st^ season	2^nd^ season	1^st^ season	2^nd^ season
**Water stress (W)**								
**I**_**0**_	42.84 a	41.78 a	15.61 a	15.24 a	9.16 a	9.42 a	4.88 ab	5.15 b
**I**_**1**_	33.37 d	32.60 d	13.27 d	12.85 d	7.57 c	7.76 c	5.06 a	5.32 a
**I**_**2**_	36.70 c	36.11 c	13.96 c	13.63 c	8.10 bc	8.58 b	4.73 b	5.16 b
**I**_**3**_	40.09 b	38.82 b	14.62 b	14.34 b	8.56 b	9.08 a	4.67 b	5.09 b
**LSD**	0.43	0.42	0.44	0.43	0.57	0.45	0.25	0.14
**Potassium application levels (K)**								
**K**_**0**_	36.66 d	35.77 d	13.84 c	13.48 c	8.16 c	8.48 b	4.81	5.14
**K**_**1**_	37.10 c	36.21 c	14.05 c	13.69 c	8.26 bc	8.59 b	4.80	5.12
**K**_**2**_	39.31 a	38.36 b	14.65 b	14.31 b	8.40 ab	8.85 a	4.85	5.25
**K**_**3**_	39.93 b	38.97 a	14.92 a	14.57 a	8.58 a	8.92 a	4.87	5.22
**LSD**	0.39	0.37	0.26	0.25	0.21	0.24	ns	Ns
**W× K**								
**I**_**0**_ **K**_**0**_	40.72 c	39.71 c	14.71 cd	14.37 cd	8.76	9.13	4.81	5.09
**I**_**0**_ **K**_**1**_	41.21 c	40.18 c	15.12bc	14.77 bc	9.06	9.07	4.87	5.01
**I**_**0**_ **K**_**2**_	44.09 b	43.00 b	16.17 a	15.79 a	9.21	9.52	4.94	5.23
**I**_**0**_ **K**_**3**_	45.35 a	44.22 a	16.43 a	16.04 a	9.62	9.95	4.91	5.26
**I**_**1**_ **K**_**0**_	31.87 i	31.14 h	12.95 i	12.54 i	7.37	7.54	5.03	5.27
**I**_**1**_ **K**_**1**_	32.31 i	31.56 h	13.04 hi	12.63 hi	7.63	7.65	5.10	5.22
**I**_**1**_ **K**_**2**_	34.39 h	33.59 g	13.47 gh	13.04 gh	7.60	7.97	5.02	5.38
**I**_**1**_ **K**_**3**_	34.91 gh	34.11 fg	13.61 fg	13.18 fg	7.66	7.90	5.08	5.42
**I**_**2**_ **K**_**0**_	35.18 fg	34.61 ef	13.73 efg	13.39 efg	7.98	8.34	4.71	5.09
**I**_**2**_ **K**_**1**_	35.73 f	35.15 e	13.84 efg	13.50 efg	8.06	8.55	4.71	5.14
**I**_**2**_ **K**_**2**_	37.85 e	37.25 d	14.08 ef	13.76 e	8.19	8.84	4.77	5.33
**I**_**2**_ **K**_**3**_	38.04 e	37.43 d	14.21 de	13.88 de	8.17	8.57	4.71	5.10
**I**_**3**_ **K**_**0**_	38.85 d	37.62 d	13.96 efg	13.64 ef	8.51	8.90	4.67	5.10
**I**_**3**_ **K**_**1**_	39.17 d	37.93 d	14.19 e	13.87 e	8.29	9.09	4.54	5.09
**I**_**3**_ **K**_**2**_	40.92 c	39.62 c	14.89 c	14.65 c	8.58	9.05	4.68	5.06
**I**_**3**_ **K**_**3**_	41.43 c	40.11 c	15.44 b	15.19 b	8.85	9.26	4.78	5.12
**LSD**	0.77	0.75	0.51	0.50	ns	ns	ns	ns

I_0_ = no stress, I_1_ = pre anthesis stress, I_2_ = anthesis stress, I_3_ = post anthesis stress, K_0_ = 0 kg K ha^-1^, K_1_ = 50 kg K ha^-1^, K_2_ = 100 kg K ha^-1^, K_3_ = 150 kg K ha^-1^, LSD = least significant difference, ns = non-significant, Mean values sharing the same letter in a column do not differ significantly at P = 0.05

RETRACTED

**Table 7:** Correlations coefficient (r) of yield components with achene yield.

Yield Components	Achene Yield	
	1^st^ Season	2^nd^ Season
Plant height	0.92***	0.94***
Head diameter	0.92***	0.91***
No. of achene’s head^-1^	0.92***	0.94***
1000 achene weight	0.93***	0.92***
Biological yield	0.97***	0.98***
Hasrvest index	0.96***	0.95***
Oil Contents	0.98***	0.97***
Protein contents	0.91***	0.92***
Nitrogen uptake	0.98***	0.96***
Phosphorus uptake	0.89***	0.90***
Potassium uptake	0.94***	0.94***

## Discussion

Water stress at different crop growth stages significantly decreased yield and yield attributes. Plant height, head diameter, number of achenes and 1000-achene weight were closely related to achene yield. Severe yield reduction in pre-anthesis stress during the spring season is primarily due to high evaporative demands.

Yield and yield components were reduced by water stress at critical stages, especially at pre-anthesis and anthesis. However, post-anthesis water stress caused less yield reduction. Pre-anthesis and anthesis stress reduce yield potential because available water at these stages is insufficient during canopy formation and reproductive development.

Better performance of sunflower in terms of yield and yield components under higher K fertilization is due to the involvement of K in main osmotic solute of plants [28, 37]. Potassium accumulation at the cellular level results in osmotic water uptake and generation of cell turgor needed for stomatal opening and plant growth [38, 39]. Potassium influx inside the stomatal guard cells cause water accumulation leading to their swelling and subsequent stomatal opening, allowing CO_2_ and transpired water vapors to move freely in and out of plant tissues. Under water stress, potassium efflux from guard cells and the pores close tightly to prevent water loss. In case of inadequate supply of K, the stomatal activity becomes slow and water losses are high. However, adequate K supply increases plant uptake of water as well as improves its use efficiency within the plant [39–41].

High K application increases leaf water content and lead to K accumulation in the vacuoles, causing stomatal uptake of water, resulting in higher cell turgor and growing cells, induces cell elongation and decreases stomatal density. It reduces daily accumulated transpiration water loss from leaves and makes the bulk leaf water relations favorable [42].

Increased K requirement in plants is due to its involvement in regulating photosynthetic CO_2_ fixation. Drought-induced impaired stomatal movement results in reduced CO_2_ fixation. Increasing severity of water stress leads to higher K demand to regulate photosynthesis and protect chloroplast against oxidative damage. Drought-induced yield reduction is greatly mitigated by increasing K fertilization [15, 42–44].

RETRACTED

Leaf area index is the major component directly related to plant growth and yield. Reduction in leaf growth decreases biomass of all other plant components. The better yields were associated primarily with the presence of more leaf area during early seed development [45]. Water stress at critical stages significantly influences sunflower growth, yield attributes, and achene quality [46, 47]. Besides affecting leaf area, pre-anthesis stress also reduces plant height [48, 49]. Like other crops, water deficit experienced during different stages of crop development in sunflower, resulted in compromised CGR, significantly contributing to the yield anomalies [50–53].

Examination of the variation in the content of the four major fatty acids (stearic, palmitic, linoleic, and oleic acid) showed that the oil fatty acid composition at the initial phases of seed formation differed substantially from matured seeds [15, 54]. Oleic and linoleic acid concentrations in oil are significantly affected by growing conditions. Water stress at anthesis and mean temperature probably affected linoleic and oleic acid concentration. However, average linoleic and oleic contents of the oil were not affected by irrigation regimes [15]. Cooler weather can extend the duration of the grain fill period; however, could alter the composition of fatty acids in the oil. Cooler temperature can slow the conversion of linoleic acid fatty acid to oleic forms in oilseed [55, 56]. Adequate water supply is required during grain filling to achieve high oil concentration [15].

Prevailing temperature during seed development has a key influence on sunflower oil characteristics [57], mainly as a result of synthesis or activation of oleate desaturase at low temperature and its reversible inhibition at elevated temperature [58, 59]. Irrigation may influence the temperature of the vegetative apparatus and the canopy micro-climate [60], increased evapotranspiration cooling of plant tissues after irrigation might have resulted in increased activity of oleate desaturase, causing a lower oleic/linoleic acid ratio [58].

The interaction of N, P, and K is widely discussed in the literature. Potassium application is vital for efficient utilization and resultant synergistic benefits of N and P application [61, 62]. The yield response to limited irrigation can be greatest if water is applied to alleviate deficits during critical growth stages of yield formation and proper fertilizer application.

RETRACTED

## Conclusion

Different growth stages of sunflower significantly varied in their response to water stress. Pre-anthesis stage proved highly susceptible to water stress in terms of plant height, head diameter, achene weight, achene yield, biological yield, and harvest index. Similarly, oil and protein contents, crop growth rate, and oleic acid concentration in seed were lowest when water stress was imposed at pre-anthesis stage. Water stress had non-significant effect on stearic acid and palmitic acid concentration. Increasing potassium level had positive effect on the studied parameters, except palmitic acid contents. Increasing potassium fertilizer level significantly helped sunflower plants to recover from water stress. The lowest values of average achene weight, achene yield, biological yield), oil contents, protein contents, uptake of nitrogen, and potassium were recorded for water stress at pre-anthesis stage without potassium application. However, values of these parameters significantly improved with increasing levels of potassium application. Normal irrigation (without stress) treatment combined with higher potasssium application (150 kg ha^-1^) resulted in the highest values for growth, yield, and quality attributes. Higher potassium requirement of sunflower during water stress conditions can be the potential reason for these results. Therefore, it concluded that better yield and quality of sunflower can be obtained under water with the application of higher rates of potassium.

## Supporting information

S1 Dataset (XLSX)
